# Transition from child to adult health care for patients with lysosomal storage diseases in France: current status and priorities—the TENALYS study, a patient perspective survey

**DOI:** 10.1186/s13023-022-02232-w

**Published:** 2022-02-21

**Authors:** Delphine Genevaz, Armelle Arnoux, Catherine Marcel, Anaïs Brassier, Samia Pichard, François Feillet, François Labarthe, Brigitte Chabrol, Marc Berger, Anne-Sophie Lapointe, Yvann Frigout, Bénédicte Héron, Gilles Chatellier, Nadia Belmatoug

**Affiliations:** 1 Vaincre les Maladies Lysosomales (VML), Massy, France; 2 Clinical Investigational Center 14-18, Clinical Epidemiology INSERM & Clinical Research Unit, Assistance Publique-Hôpitaux de Paris Centre, Paris University & European Hospital Georges Pompidou, Paris, France; 3 Reference Center for Lysosomal Diseases, Assistance-Publique Hôpitaux de Paris, Beaujon Hospital, Paris University, Paris, France; 4 Reference Center for Inherited Metabolic Diseases, Assistance Publique-Hôpitaux de Paris, Necker Hospital, Paris University, Paris, France; 5 Reference Center for Inherited Metabolic Diseases, Nancy University Hospital, Vandoeuvre-lès-Nancy, France; 6 Reference Center for Inherited Metabolic Diseases, Clocheville Hospital, University Hospital, Tours, France; 7 Reference Center for Inherited Metabolic Diseases, Assistance Publique-Hôpitaux de Marseille, University Hospital of Marseille, Marseille, France; 8 Reference Center for Lysosomal Diseases, Estaing University Hospital, Clermont Ferrand, France; 9 Reference Center for Lysosomal Diseases, Assistance Publique-Hôpitaux de Paris, Trousseau Hospital, Sorbonne University, Paris, France

**Keywords:** Lysosomal diseases, Transition from childhood to adulthood, Patient survey, Patient opinion

## Abstract

**Background:**

Transition from childhood to adulthood (TCA) is usually difficult in rare, progressive and multisystemic diseases. New treatments and modalities of care for many lysosomal diseases (LD) can increase life expectancy, and a successful TCA can help patient who reach adulthood to avoid disruption to health care. In France, some TCA initiatives have been taken by referral centers but in view of the problems encountered by *Vaincre les Maladies Lysosomales* (VML), the LD patient association, they seem to be insufficient. The aim of this study is to determine the current state of the TCA process and to identify actions to improve it through interviews with patient families and physicians in LD referral centers. The study is based upon an observational, non-interventional, cross-sectional, national survey which used two anonymous questionnaires. These questionnaires, developed by a scientific committee including representatives from VML and medical specialists in LD, were sent to patients who were receiving care in pediatric departments at age 15 years or older. Questionnaires were also sent to their referral pediatricians.

**Results:**

Fifty-four patients were included. Forty-two questionnaires were completed by patients and their corresponding physicians and 12 were completed by physicians only. The majority of the patients (80%) were informed that transfer to adult healthcare would occur, but 52% were informed after their eighteenth birthday. Forty-eight percent indicated that they were informed that a TCA coordinator would be appointed; for 39% the time frame for the transfer was communicated, and 31% were informed of the composition of the adult medical team. Among the actions that patients rated as “important/very important”, and considered to be a priority in their comments, the most frequently cited were the provision of explanatory documents on the TCA (94%), the transmission of the medical file from the pediatric sector to the adult sector (94%) and a joint consultation with both pediatrician and adult unit physician (91%). Physicians were in agreement concerning the primary importance of the last two actions.

**Conclusion:**

This study provides a basis for the deployment, on the national level, of transition programs which include specific actions that patients view as priorities.

## Background

In recent years, programs to facilitate the transfer of patients from pediatric to adult care for diseases such as diabetes [1, 2], inflammatory rheumatisms, congenital heart diseases and rare liver diseases [3] have been implemented and are regularly evaluated and optimized. They include recommendations for action and have been approved by medical societies and regulatory authorities [4]. Similarly, in rare diseases, transition issues are increasingly being explored and identified, as well as factors which are favorable or unfavorable to a successful transition [5–8]. This has led to the creation and implementation of genuine transition programs, for example in cystic fibrosis, sickle cell disease, celiac disease, rare neurological diseases and juvenile arthritis, thus helping to optimize patients’ health status and continuity of care and to improve compliance and monitoring [9–11].

Like many other rare diseases, lysosomal storage diseases are multisystemic, chronic, heterogeneous and progressive, and most of them are very disabling. In recent years the evolution of care has allowed more patients to reach adulthood—improved diagnosis, patient care, treatments, awareness-raising by expert referral centers and better policies with regard to rare diseases have all contributed to this outcome. As a result, physicians treating adults are increasingly confronted with serious, rare diseases with which they may have little or no familiarity. This development requires action to ensure appropriate transition programs.

Regarding lysosomal storage diseases, specific initiatives and procedures based on current status and recommendations [12–14]*,* have been set up by some referral centers to improve transition. These include multidisciplinary consultations involving pediatricians and physicians for adults; awareness-raising for physicians treating adults during medical congresses; and improved efficiency in the transfer of medical records. The need to organize transition is mentioned in France in the National Protocols for the Treatment of Rare Diseases (PNDS) [15] and on the European level, in the European Rare Disease Networks (ERN: European Reference Networks). Nonetheless*,* the French patient association *Vaincre Les Maladies Lysosomales* (VML) continues to be contacted by patients and families with regard to practical hurdles and difficulties created by organizational deficiencies, poor information and lack of knowledge concerning the transition process.

In light of these difficulties, VML and the referral center for lysosomal storage diseases designed the national survey TENALYS (transition to adult care in lysosomal storage diseases). The objective of the TENALYS survey was to gather information from patients on existing transition practices and their opinions about these practices, to identify priorities, and to obtain views from pediatricians concerning actions to improve the transition.

## Methods

### Study design

This is an observational, non-interventional, cross-sectional national survey. Two different anonymous questionnaires were used: one completed by patients with lysosomal storage diseases (or parents), and another by a physician at the pediatric center providing care to the patient.

### Population

#### Inclusion criteria

The survey was designed for patients meeting three conditions: (i) aged 15 or older; (ii) a lysosomal storage disease diagnosed before adulthood; (iii) disease management in a pediatric department.

#### Exclusion criteria

Patients whose clinical condition contraindicated transition to an adult department at the time of the survey, according to the pediatric center physicians’ opinion, were excluded from consideration, as were patients who were taking part in clinical trials.

### Research protocol

The project was designed by a Scientific Committee composed of physicians from the Lysosomal Storage Disease Reference Center, as well as the President and the Scientific Officer of VML.

The participating pediatric centers were the referral centers for hereditary metabolic diseases, together with some local pediatric hospitals caring for patients with lysosomal storage diseases. The centers were contacted by mail. The study documents were then sent to investigators who agreed to participate and to provide the consent form and questionnaire to their patients (or their patients’ parents). Investigators and patients (or parents) returned the completed questionnaires directly to the clinical research unit responsible for processing the data, regulatory management, study logistics, data management, statistical analysis and storage (CIC1418—CE, INSERM & Clinical Research Unit Assistance Publique-Hôpitaux de Paris).

### Data management/data questionnaire collection

The patient questionnaire was prepared and developed by the Scientific Committee on the basis of evidence obtained by the patient association from patients and families. A trial questionnaire was evaluated by 10 young adult patients (or parents) who had already experienced the transition to adult care and evaluated for comprehensibility, quantity of questions and completion time. The questionnaire for physicians in the pediatric investigation centers was modelled upon the patient questionnaire.

The main sections of both questionnaires concerned the socio-demographic characteristics of the patient, the disease, its functional impact, and patient management. The questionnaires also included open questions on the transition process in which respondents were invited to identify the most important actions. The patient questionnaire also included closed questions about transition preparation, transition information, and the organization of the transition. For each item, the patient (or parents) was asked to specify whether certain actions had been taken or not and to rank the importance of each action.

Paper questionnaires were entered twice at the clinical research unit, by two independent people for prevention of typographical errors prior to data recording and storage into a PostgreSQL database. Each patient was assigned a unique code number combined with his/her initials. The patient identification code lists permitting identification of patients from their ID were kept only by sites where patients have been enrolled. Neither the sponsor nor the data processor has an access to these lists

### Statistical analysis

A preliminary analysis of the active patients monitored in pediatric referral centers showed that data collection from a sample of 60 patients was feasible.

The questionnaires completed by the pediatric investigators served as the basis for the description of the patient population included in the study.

The questionnaires completed by patients (or parents) were used to describe what is done in practice regarding preparation, information, and the organization of the transition, and to determine the importance of each process.

Actions that appear to be priorities to facilitate the transition were described by both patients (or parents) and pediatric investigators in the respective questionnaires.

For the analysis of the responses to the open questions, the Scientific Committee drew up a list of 17 potential terms beforehand. Comments collected from investigating physicians and patients (or parents) were compared with this list, either to add missing terms or to reduce the list (remove unnecessary terms).

The results of the statistical analyses are provided with a number (n) and a proportion (%).

Bivariate analyses for group comparison were performed on the answers provided by patients (or parents) in the questionnaires to explore factors contributing to the absence of a transition at 21 years of age. This threshold was imposed by the fact that 21 is the age limit for care in French pediatric facilities, even though legal majority is reached at age 18. Chi-square tests and Mann-Whitney tests were used for qualitative and quantitative factors respectively.

The data was analyzed using SAS 9.4 software (SAS Institute Inc., Cary, NC, USA).

### Regulatory authorizations

The study obtained all regulatory authorizations (opinion of the Advisory Committee on the Processing of Healthcare Information—CCTIRS) and a favorable rating from the ethics committee (CPP Île de France II # 2015-05-06). The research was conducted in the investigation centers in accordance with the Declaration of Helsinki and the GCP in force.

## Results

Thirty nine pediatric centers (16 pediatric referral centers for inherited metabolic diseases and lysosomal storage diseases and a sample of 23 local pediatric hospitals) were contacted. Fourteen of them agreed to participate. Ultimately, 7 pediatric investigation centers (one investigator for each center), all referral centers for inherited metabolic diseases, participated in the survey.

Fifty-five patients (or parents) gave their written consent to the investigators to participate in the survey but only 54 were analysed (one patient was excluded because he/she was participating in a clinical trial). Forty two patients (78%) actually returned their questionnaire directly to the clinical research unit once completed. Investigators completed on their side a questionnaire for each participating patient (54 questionnaires). The description of patient characteristics was based on 54 questionnaires completed by 7 investigators. The analyses of the 42 questionnaires completed by patients, described existing transition practices, opinions about these practices and identified priority TCA actions. The prioritization of TCA actions according to the pediatric investigators, was provided by the investigators questionnaires.

### Patient characteristics

Patients’ demographic and clinical characteristics and distribution according to age (younger or older than 21 years) are described in Table 1. This information came from the 54 questionnaires completed by the pediatric investigators.

**Table 1:** Characteristics of patients monitored in a pediatric department

Characteristics	Patients Overall n = 54	Patients ≥ 15 < 21 years old n = 41	Patients ≥ 21 years old n = 13
Gender, male n (%)	34/54 (63.0%)	23/41 (56.1%)	11/13 (84.6%)
Disease			
Mucopolysaccharidosis	35/53 (66.0%)	25/41 (61.0%)	10/12 (83.4%)
Gaucher type 1	6/53 (11.3%)	5/41 (12.2%)	1/12 (8.3%)
Alpha mannosidosis	3/53 (5.7%)	3/41 (7.3%)	–
Fucosidosis	2/53 (3.8%)	2/41 (4.9%)	–
Metachromatic leukodystrophy	2/53 (3.8%)	1/41 (2.4%)	1/12 (8.3%)
Others (Fabry, gangliosidosis, Danon, cholesteryl ester storage disease, Niemann-Pick type B: n = 1 each)	5/53 (9.4%)	5/41 (12.2%)	–
Other patient characteristics			
Chronic pain	18/52 (34.6%)	14/40 (35.0%)	4/12 (33.3%)
Orthosis need	8/51 (15.7%)	8/39 (20.5%)	0/12 (0.0%)
Mechanical respiratory	12/53 (22.6%)	10/40 (25.0%)	2/13 (15.4%)
Mobility assistance	23/54 (42.9%)	20/41 (48.8%)	3/13 (23.1%)
Disability*	40/54 (74.1%)	30/41 (73.2%)	10/13 (76.9%)
Hospitalization or surgery in the last 6 months or planned in the next 12 months	14/54 (25.9%)	13/41 (31.7%)	1/13 (7.7%)
Treatment by/for			
Enzyme replacement therapy	34/53 (64.1%)	25/41 (61.0%)	9/12 (75.0%)
Epilepsy	10/54 (18.5%)	9/41 (21.9%)	1/13 (7.7%)
Sleeping disorders	4/54 (7.4%)	4/41 (9.7%)	0/13 (0.0%)
Spasticity	2/54 (3.7%)	1/41 (2.4%)	1/13 (7.7%)
Tremor	2/54 (3.7%)	2/41 (4.8%)	0/13 (0.0%)
Transplantation:	9/53 (17.0%)	7/40 (17.5%)	2/13 (15.4%)
Heart	1/9 (11.1%)	1/7 (14.3%)	0/2 (0.0%)
Bone marrow	8/9 (88.9%)	6/7 (85.7%)	2/2 (100.0%)

*Difficulty with at least one of the following: hearing/sight/speech/writing/attention/memory/learning/comprehension

### Questionnaire results concerning TCA preparations

#### Patient questionnaires: current status

In 12% of cases, questionnaires were completed by patients alone, 43% were prepared with parental assistance, and 28% by parents alone. Data were missing in 17%. Information knowing who completed the questionnaire was not provided in 17%. The analysis of the 42 questionnaires completed by the patients (or their parents) revealed that 33/41 patients (80%) had been informed that a transfer from pediatric to adult health care would occur (data for this item was missing data in one questionnaire). Among the 33 patients who received such information, 17/33 (52%) had been informed after they reached adulthood (18 years), including the 8 patients over 21 years old. In the subgroup of patients informed that a transfer would occur (n = 33 patients), answers about the main TCA actions proposed to patients are described in Fig. 1A.

**Fig. 1:** **A** Patient’s responses on proposed actions and priorities for TCA, **B** Physicians’ responses on priorities for TCA

#### Importance of TCA actions according to patients (or parents)

With reference to a proposed set of actions for a TCA (Fig. 1A), we note that 10% of patients (or parents) reported receiving background documents explaining the TCA, an action ranked as important/very important by the most patients (94%). Joint consultations involving the pediatrician and the physician for adults were rarely proposed (6%) whereas 91% of patients considered them to be important/very important.

Only 6% of patients reported receiving their medical records for the TCA whereas 87% considered it important/very important to receive them.

Questionnaires included an open question asking respondents what they considered to be the most important actions facilitating a TCA. Twenty-four patients replied (57%). Two actions were particularly reinforced: the transfer of medical record (33%) and joint consultations (29%). An additional desired action was added: find a trained, skilled and efficient staff in the adult department.

#### Comments of pediatricians on TCA priorities

For pediatric investigators (6/7), the principal actions needed to facilitate a smooth TCA, were (i) joint consultations with pediatricians and adult department physicians and (ii) the anticipation and progressive preparation of the TCA through information provision. The third most important action (5/7) mentioned was “the efficient organization of the adult unit, the assurance of availability of treatment, and multidisciplinary consultations” (Fig. 1B).

#### Reasons for continuing care in pediatric departments after the age of 21

Thirteen patients were over 21 years old at the time of inclusion. Queried about the rationale for continued care for these patients in a pediatric setting, pediatric investigators explained that the transition was actually underway for 4 patients. For 7 patients, the reasons provided were (i) lack of TCA organization (n = 3); (ii) lack of knowledge about the disease on the part of physicians for adults (n = 2); (iii) refusal of transfer to adult medicine on the part of the family or patient (n = 2), (iv) TCA not proposed (n = 1). Answers were missing in two questionnaires.

Nine questionnaires were returned by patients over 21 years old. Only 4 of them gave the reasons why they were still in pediatric care. The causes mentioned were (i) a lack of organization in the adult medicine department (n = 3) and (ii) refusal by the family or patient (n = 1).

#### Potentially unfavourable circumstances for TCAs

During the analysis of the results, we hypothesized that a TCA could be more complex/difficult when illness was severe or when the patient was over 21 years of age, situations which would justify retrospective bivariate analyses. To test this hypothesis, we compared (i) patients with MPS (the population most represented in the study) with other lysosomal storage diseases, (ii) patients with a neuro-cognitive disorder with absence of these disorders, (iii) patients with difficulties in at least one of the following areas: hearing/sight/speech/writing/attention/memory/learning/comprehension with patients without such difficulties, (iv) patients over 21 years of age with those under 21 years of age. These comparisons did not reveal any significant factors related to health status or management in our study population.

## Discussion

It is particularly important that pediatric services in rare disease referral centers have effective programs for transition to adult care, adapted to the diseases and patients for whom they provide care. As has already been found in other countries, the tasks and missions involved in transition are numerous and can sometimes be difficult to carry out [12, 14, 17]. In order to achieve optimal results for patients with lysosomal storage diseases, we reviewed current practices in pediatric units where these patients are followed, identifying the actions that seemed most important from the point of view of the patients (or their parents) and the pediatricians responsible for their care.

Our review indicates that most patients had well been informed that, at some point, there would be a transfer from pediatric units to adult medical care. In almost half of the cases under consideration, some practices which facilitate transition were already in place, such as the designation of a transition coordinator and the provision of information about the timing of the transfer. Other practices were encountered less frequently, such as the provision of information about the composition of the adult medical team, organizing an appointment with the pediatrician alone, without the parents’ presence, and forwarding medical records from the pediatric to the adult medical unit. Other initiatives, such as having patients visit the adult unit, producing explanatory documents about the transition and organizing joint consultations with the pediatric and adult teams, are not widespread.

Some centers do implement the practices that the majority of patients consider to be important/very important. In view of the expectations and preferences expressed by the patients in this survey, their systematic use by healthcare teams can be recommended.

Patients (or their parents) consistently prioritize the provision of explanatory documents about the transition. These documents must be readily available and comprehensible for both patients and caregivers.

Patients and physicians agree on the importance of forwarding the medical records from the pediatric department to the relevant adult unit and of the organization of joint consultations with both pediatric and physicians for adults, even if organizing actual appointments can be challenging (different geographic areas, different availability, uncertainties regarding reimbursement). The French hereditary metabolic disease network (G2M) is currently developing a transition document equivalent to the transition health passport developed by certain participating teams. This kind of document including information from the pediatric record, treatments, risk situations, the most recent pediatric examinations, social, educational and professional considerations, and follow-up elements, could be in accordance with the patient’s expectation.

Although rarely mentioned by physicians, patients emphasized the importance of a coordinator responsible for preparing the necessary documents, organizing the care process and setting up of meetings between patients (with or without the parents) and both the pediatric and the adult care teams. The coordinator can also help inform and train the future paramedical team.

For more than half of the patients, information on the timing of the transfer was provided belatedly, after the age of 18 years. It is important to anticipate the TCA, to mention it early and often, and to explain that it will only take place once the disease has been stabilized and never during an acute medical event. Transition is the gradual process that leads to the actual transfer of care. A date cannot always be set with precision and may be subject to change. This must be reiterated throughout the transition process.

Patients and, to a lesser extent, physicians in the pediatric centers would like to be familiar with the composition not only of the adult medical team but also the paramedical team and the adult department units. At the same time, the physicians who provide care to these patients in pediatric settings often have difficulty identifying referral physicians in the future adult medical department. All these unknowns (date, teams, locations) often generate stress and anxiety for patients and their families but also for pediatric physicians in charge of the transition.

Social networking and exchanges of general information about the TCA do not appear to be important for most patients/parents (23.3%), who seem to prefer personal discussions with a view to obtaining practical information specific to their situation.

Responses concerning consultations with or without parents are relatively difficult to interpret because, most often, the questionnaires were completed by the parents. Their responses may reflect a fear that if their child is alone with the physician, they will not share enough information about their medical history. Physicians from adult departments are less accustomed to the presence of parents, who can often provide significant help through their knowledge and experience of the rare disease and the patient’s experience. On the other hand, consultation time alone with the patient is essential when more personal subjects such as sexuality or possible addictions are addressed. The best approach is undoubtedly case-by-case.

The principal concerns expressed by pediatric physicians relate to (i) the experience, competence, and organization of care on the part of the adult medical and paramedical team, (ii) the possibility of multidisciplinary consultations, (iii) the availability of drugs and equipment adapted to patients’ disabilities.

As noted, improved understanding and management of lysosomal storage diseases in childhood have led to an increase in the number of patients entering adulthood. At the same time, few adult care physicians have been trained in the management of lysosomal storage diseases. To avoid disruption of care it is therefore essential to train coming generations of physicians and paramedical staff from the adult unit in the care and management of these diseases.

By definition, rare diseases do not allow for the recruitment of large research samples, and the number of participating patients is a limiting factor with respect to the statistical power of possible post-hoc statistical analyses. In France, lysosomal storage disease management generally takes place in referral centers. Nine pediatric centers did not include patients for various reasons (lack of time, refusal, no target population). Some patients, especially the least symptomatic, are followed in hospitals scattered throughout the country. Therefore, no pediatric centers close to patients’ homes participated in the study. It is possible that these centers did not have time to identify and include patients, or that they felt less comfortable with academic studies on medico-social themes.

In the complementary exploratory analyses, the comparison of patients over 21 years of age with those under 21 years of age did not reveal any factors explaining why these patients remain in pediatric care. Given the population size, these analyses suffer from a lack of statistical power.

The strength of the study lies in the long-standing professional relationships between VML and the Lysosomal Storage Disease Reference Center. These relationships made possible a dialogue through which common TCA problems could be identified.

In this study, the population size is sufficient to describe accurately the current status of TCA in the participating centers. The patient questionnaire return rate of 78% is satisfactory and similar to a telephone call-back study [16]. The closed questions were developed and tested in a pilot phase, using qualitative questionnaires and interviews with 10 patients or parents who had undergone the transition. Moreover, the existence of comment fields allowed for the provision of very informative additional information, which most often supplemented the answers to closed questions. By citing existing actions and their impact, this study helped TCA stakeholders define their needs and priorities. This review of TCA practices underscores the need expressed in the 3rd Rare Diseases Plan [17]: priorities identified should be integrated into and funded under therapeutic education programs and projects for organizing the improvement of care systems in France.

Based on the TENALYS study, our network is implementing actions organized by a designated coordinator to:

- improve communication on the TCA for patients and parents by developing more documentary resources;
- anticipate the transfer of the medical record and all useful knowledge concerning the patient’s medical history;
- create a patient document follow-up on TCA, easily available for all actors involved in the care of the patient;
- increase and improve joint consultations in dedicated and adapted spaces by organizing multidisciplinary team mobility.

## Conclusion

In this study, the needs expressed by patients with lysosomal storage diseases are clear. We consider it essential for all healthcare staff in referral centers caring for these patients to increase efforts to meet their expectations, with reference to a set of priority actions for improvement. Three actions have been shown to be particularly important. The first is to provide patients with background documents which explain the TCA. The second action, desired by both patients and pediatric physicians, is the forwarding of the medical records, or a summary thereof, from the pediatric service to the adult unit. The third action consists in the organization, preferably by a designated coordinator, of a joint consultation bringing together the patient, the pediatrician and the adult care physician.

A supplementary study of adult patients who have recently completed their TCA could be usefully undertaken to further elucidate conditions making for successful transfers.

## Data Availability

The data that support the findings of this study are available on request from the corresponding author NB. The data are not publicly available due to information contained in the database could compromise research participant privacy/consent.
